The article "Computational Analysis of the Pulmonary Arteries in Congenital Heart Disease: A Review of the Methods and Results" was published in 2021. Journal: Comput Math Methods Med.

# Computational Analysis of the Pulmonary Arteries in Congenital Heart Disease: A Review of the Methods and Results

**DOI:** 10.1155/2021/2618625

**Published:** 2021-04-01

**Authors:** M. Conijn, G. J. Krings

**Affiliations:** Pediatric Cardiology, Wilhelmina Children's Hospital (University Medical Center), Utrecht 3584 EA, Netherlands

## Abstract

With the help of computational fluid dynamics (CFD), hemodynamics of the pulmonary arteries (PA's) can be studied in detail and varying physiological circumstances and treatment options can be simulated. This offers the opportunity to improve the diagnostics and treatment of PA stenosis in biventricular congenital heart disease (CHD). The aim of this review was to evaluate the methods of computational studies for PA's in biventricular CHD and the level of validation of the numerical outcomes. A total of 34 original research papers were selected. The literature showed a great variety in the used methods for (re) construction of the geometry as well as definition of the boundary conditions and numerical setup. There were 10 different methods identified to define inlet boundary conditions and 17 for outlet boundary conditions. A total of nine papers verified their CFD outcomes by comparing results to clinical data or by an experimental mock loop. The diversity in used methods and the low level of validation of the outcomes result in uncertainties regarding the reliability of numerical studies. This limits the current clinical utility of CFD for the study of PA flow in CHD. Standardization and validation of the methods are therefore recommended.

## 1. Introduction

Stenosis of the pulmonary arteries (PA's) is commonly seen in patients with congenital heart disease (CHD). It can occur as a native substrate or after surgery [1]. Diagnosing patients with PA stenosis can be challenging as cardiac echography may be inconclusive. To confirm the diagnosis, often evaluation with multiple imaging modalities as CTA and CMR is necessary. The decision whether to treat the stenosis is primarily based on pressure gradients which need to be confirmed by cardiac catheterization [2]. However, pressure gradients might resolve under anesthesia resulting in possible under treatment of PA stenosis. In addition, restenosis and intima proliferation can occur after treatment. The mechanisms causing this are still not well understood, but several flow characteristics—i.e., turbulence, wall shear stress (WSS), and the interaction of flow and (stent) geometry—are hypothesized to be of influence [3–5]. Computational fluid dynamics (CFD) provides the opportunity to study these factors and enhance our knowledge of hemodynamics in the PA's. It allows for detailed flow visualization and simulation of exercise and treatment outcomes. However, its clinical use is still limited as there is a great variety in used methods and validation of the numerical outcomes is often challenging [6–11]. The aim of this review was to analyze the available literature on numerical studies of the pulmonary arteries in biventricular CHD, focusing on the used methods and validation of the results.

The article "Computational Analysis of the Pulmonary Arteries in Congenital Heart Disease: A Review of the Methods and Results" was published in 2021. Journal: Comput Math Methods Med.

## 2. Methods

### 2.1. Search Strategy

A PubMed and Embase search was performed. The searched papers needed to include “pulmonary arteries” and “computational fluid dynamics” or a synonym in their title or abstract. The language for the search was restricted to English. All papers published before 1^st^ of January 2021 were included.

### 2.2. Inclusion and Exclusion Criteria

All papers on numerical analysis of the PA's in biventricular hearts were included. Pediatric and adult as well as animal studies were considered. Papers with the focus on pulmonary hypertension were excluded as well as papers from before 2001, reviews, and if no full text was available. All inclusion and exclusion criteria are shown in Figure 1.

## 3. Results

### 3.1. Study Selection

The search in the PubMed and Embase databases resulted in a total of, respectively, 266 and 286 papers. After undoubling and title abstract screening, 45 papers remained. The full-text screening of these papers revealed exclusion criteria for 11 articles. This resulted in a total of 34 eligible papers for this review. The flowchart for the selection process is shown in Figure 1.

### 3.2. Study Overview

The 34 selected papers included four animal studies and 25 papers presenting human cases. In one paper, both human and animal cases were described [12]. In six studies, PA's were represented by straight or curved tubes [13–18]. Altogether, the articles presented a total of 256 geometries based on 126 subjects (Table 1).

Over half of the included papers focused on the surgical treatment of PA stenosis. These 19 studies described the use of CFD in surgical planning, for comparison of different shunt configurations or to study (post)surgical complications [13–16, 18–31]. In two papers, numerical studies were used to evaluate interventional strategies [32, 33]. One of these described a CFD-assisted patient-specific stent design for PA interventions, and the other studied a new device for percutaneous pulmonary valve replacement. Technical strategies for CFD analysis were the main subject in five papers [12, 34–37]. The focus was on improving or simplifying the process of numerical modeling of the PA's. The remaining eight papers described hemodynamics in the PA's, for example, comparing rest and exercise conditions or describing the hemodynamic impact of abnormal anatomy [17, 37–43].

The article "Computational Analysis of the Pulmonary Arteries in Congenital Heart Disease: A Review of the Methods and Results" was published in 2021. Journal: Comput Math Methods Med.

Of the 34 studies, 13 were published in journals with a clinical orientation [13, 16, 18, 20–22, 25, 27–30, 37, 43]. Most of these papers—nine, respectively—were published in cardiovascular surgical journals [13, 21, 22, 25, 27–30, 43]. The other 21 studies were published in technical journals, for example, focusing on biomedical engineering or numerical methods in medicine [12, 14, 15, 17, 19, 23, 26, 31–42, 44].

In the following sections, the various used methods for numerical analysis of the PA's will be compared. The sections are subdivided into the major steps necessary for solving a CFD case. First is the anatomic reconstruction, then the meshing and setting the boundary conditions followed by the numerical setup and finishing with postprocessing and validation of the results.  Table 2 provides a summary of the different strategies used in the selected papers.

### 3.3. (Re)construction of the Geometry

Figure 2 shows the source for reconstruction of the geometry used in the selected papers. In 23 of the 34 papers, at least one patient-specific anatomy was reconstructed. The source for this reconstruction was a cardiac CT in 16 studies and CMR in six studies [12, 18, 20, 21, 23, 25, 26, 30–37, 39–45]. In the remaining two studies, multiple plane measurements on cardiac angiography were taken after which the anatomy was reconstructed [16, 27]. For surgical studies, often, one patient-specific anatomy was created after which the anatomy was altered to mimic various surgical approaches.

Most groups (re)constructed a geometry consisting of the main PA bifurcation and the right and left pulmonary artery [17, 18, 21, 22, 28, 29, 32–34, 38–40]. All these models had one inlet and two outlets. Shunt anatomy was mostly represented by one aortic or shunt inlet and two or three outlets representing the RPA, LPA, and/or the descending aorta [14–16, 23, 25–27, 31, 42, 44]. In three studies, the flow in the main PA was computed using a model with one inlet and one outlet [13, 19, 20]. Kong et al. analyzed a model with one inlet and 274 outlets, making it the biggest PA anatomy studied [36]. In seven other studies, the pulmonary circulation was reconstructed up to the peripheral arteries. Here, imaging resolution was always the limiting factor for reconstruction [12, 30, 35, 37, 41, 43, 45]. The number of outlets in these studies varied between 8 and 100 outlets per model.

An artificial geometry was used in ten studies [13–15, 17, 19, 24, 28, 38]. A geometry was constructed based on general values obtained by literature or measurements in multiple patients in seven papers [17, 19, 22, 24, 28, 29, 38]. The other three studies analyzed arteries represented by ideal (curved) tubes [13–15].

The article "Computational Analysis of the Pulmonary Arteries in Congenital Heart Disease: A Review of the Methods and Results" was published in 2021. Journal: Comput Math Methods Med.

After geometry reconstruction, inlet and outlet extensions were added in four of the 34 studies [19, 21, 30, 40]. The extension of the inlet varied between five and 20 times the diameter of the inlet. The outlet region was extended 20 times the diameter of the outlet. In the other 30 studies, the inlet and outlet regions were not extended.

A variety of software was used for segmentation of the patient-specific anatomies. The most mentioned open-source software package was SimVascular (http://simvascular.org). For commercial software, this was MIMICS (Materialise, Leuven, Belgium). Other software for segmentation included ITK-SNAP (open-source, http://itk-snap.org), OsiriX (commercial, Pixmeo SARL, Geneva, Switzerland), and CardioViz3D (open-source, Asclepios Research Project, Inria Sophia Antipolis, Greece).

### 3.4. Meshing

The meshing process was—partly—described in 27 of the 34 papers, while in seven, this information was completely missing. A nonstructured meshing strategy with tetrahedral elements was used in 20 of the 27 studies [12, 14, 16, 17, 19, 21, 23, 24, 30–33, 35, 36, 39–44]. A structured mesh was applied by six groups [15, 20, 22, 28, 29, 38]. Boundary layers were described by 16 authors, but the majority of the studies did not mention any boundary layer use. Of the 27 articles specifying their meshing process, 20 reported the program they used [14, 15, 17–24, 28–30, 32, 33, 36, 39–41, 43]. In most cases, this was ANSYS software (ANSYS Inc., Canonsburg PA, USA).

A mesh independence test to evaluate mesh quality was performed in 16 of the 34 papers [14–16, 18, 19, 23, 24, 31, 33, 38–44]. In 12 of these, information on the criteria for mesh independency was provided [14, 18, 19, 23, 24, 31, 33, 38–41, 44]. These criteria included velocity profiles on different locations and a difference of <5% in calculations of pressure, velocity, or WSS. In 18 of the 34 papers, a mesh independence test was not performed or at least not mentioned. Three studies applied an element size determined by a mesh independence test performed on a different geometry [17, 21, 30]. The number of elements for the final mesh varied between 30.000 and 4 million.

### 3.5. Boundary Conditions

#### 3.5.1. Inlet

Table 3 shows all the used inlet and outlet boundary conditions in the included papers. The inlet boundary conditions were pulsatile in 23 and constant in 11 papers. The most common inlet boundary condition was flow rate (l/min) followed by velocity and pressure in 18, 10, and four studies, respectively. In two studies, an electrical system was applied at the inlet [14, 26]. The inlet conditions were patient-specific in seven papers [12, 16, 27, 39–41, 43]. In these studies, the stroke volume as well as the waveform was patient-specific. These conditions were mostly obtained by MRI or invasive measurements during cardiac catheterization. In five studies, a patient-specific stroke volume was implemented but with a general waveform [25, 30, 32, 37, 45]. This waveform was scaled to a cardiac index suitable for the analyzed geometry. In the other 23 studies, a general inlet boundary condition was used.

The article "Computational Analysis of the Pulmonary Arteries in Congenital Heart Disease: A Review of the Methods and Results" was published in 2021. Journal: Comput Math Methods Med.

In 13 papers, the applied velocity profile was specified. This was a flat or plug flow velocity profile in six and a parabolic profile in three studies [12, 16, 17, 19, 22–24, 28, 34]. Three articles implemented a Womersley flow at the inlet, and one study used a patient-specific velocity profile obtained by phase-contrast MRI [32, 39–41]. However, most studies did not mention the kind of velocity profile they used on their inlet.

#### 3.5.2. Outlet

The most applied outlet boundary condition was a constant pressure outlet. 14 studies used a variation of this condition, i.e., atmospheric pressure, zero pressure, or the mean PA or aortic pressure obtained by cardiac catheterization [15, 16, 18–22, 25, 27–30, 39, 43]. In one study, a pulsatile pressure on the LPA outlet was implemented while a Womersley velocity profile was set on the RPA outlet [40]. In another study, the outflow boundary condition was defined by the LPA : RPA flow split [42]. In five papers, the three-element Windkessel model was imposed to the outlet [32–34, 37, 45]. The pure resistance strategy was used in five studies [23, 24, 31, 41, 44]. Spilker et al. described a method for the impedance boundary condition in which they reconstructed a one-dimensional (1D) anatomy and calculated the impedance value for the pulmonary anatomy [12]. One study applied multiple outlet boundary conditions and compared results. These included zero pressure, constant pressure, prescribed flow split, and a lumped parameter model [17]. In two papers, the outlet boundary conditions were not specified [13, 38].

Patient-specific information was used to calculate resistance and Windkessel values in four papers [16, 27, 31, 32, 37, 40, 41, 45]. For this, i.e., the flow split derived from flow perfusion scans, pressure from catheterization, and cardiac output from catheterization or echocardiography were taken. The other authors estimated values based on more general information.

### 3.6. Vessel Wall Compliance

In nine of the included papers, FSI was used to simulate deformation of the vessel wall during the cardiac cycle [12, 14, 15, 19, 20, 32, 35, 37, 45]. One of these groups applied case-specific compliance [20]. Here, the mesh was subdivided in five regions. Young's modulus for each region was obtained by stretch testing the tissue of freshly harvested porcine pulmonary roots. These values were then imposed to the in silico geometry of the porcine pulmonary roots. No studies were available using patient-specific compliance in human cases. The eight other groups assumed a global and constant value for the compliance of the artery wall. The highest Young modulus was 5∗10*e*7 Pa, and the lowest 2.6∗10*e*5 [19, 32]. One group implemented a Young modulus varying between 2.6 and 4.2∗10*e*5 Pa [37]. They tuned the value until the computed outcomes matched the desired patient-specific outcomes. The wall thickness was assumed to be between 0.5 and 1.5 mm. In one article, a variable thickness of 10% of the diameter of the vessel was applied [14]. Four articles specified the Poisson ratio used. These were, respectively, 0.42, 0.45, 0.49, and 0.5 [14, 19, 35, 37].

The article "Computational Analysis of the Pulmonary Arteries in Congenital Heart Disease: A Review of the Methods and Results" was published in 2021. Journal: Comput Math Methods Med.

### 3.7. Numerical Setup

The program most used for solving the numerical cases was ANSYS Fluent (ANSYS Inc. Canonsburg PA, USA). This software package was utilized by 12 groups included in this review [16, 18, 19, 21, 23–25, 27, 30, 40, 42, 44]. Other mentioned software included CFD-ACE + (ESI group, Paris, France) and SimVascular (http://simvascular.org) and ABAQUS (Simuleon, ‘s-Hertogenbosch, the Netherlands). Four groups calculated their solution with special build-in-house software [12, 14, 35, 36]. In nine papers, the software was not specified [13, 26, 31, 33, 34, 37, 41, 43, 45].

#### 3.7.1. Fluid Characteristics

In 29 of the 34 included papers, blood was assumed to behave as a Newtonian fluid while in one paper, it was assumed to be a non-Newtonian fluid [40]. Three papers did not specify the assumption they made [13, 34, 37]. In most studies, the blood density was set to be 1060 kg/m^3^. Only three studies assigned a different density of 1050 kg/m^3^ and 1000 kg/m^3^, respectively [33, 35, 40]. In nine papers, the used density was not described. Viscosity was mostly assumed to be 0.004 kg/ms [12, 14, 15, 17, 21, 22, 28–30, 33, 39, 41, 42, 45]. Other imposed values were 0.0035 kg/ms, 0.003 kg/ms, and 0.00371 kg/ms [25, 26, 35, 38, 43, 44]. Four authors applied a varying viscosity number [16, 18, 36, 40]. One of them varied the viscosity of blood between 0.003 and 0.008 kg/ms depending on hematocrit levels varying between 30 and 55% [16]. Two authors used the Carreau model to capture the varying viscosity of blood depending on the shear rate [18, 40]. The last one analyzed the stability of their algorithm with varying viscosity numbers [36].

The article "Computational Analysis of the Pulmonary Arteries in Congenital Heart Disease: A Review of the Methods and Results" was published in 2021. Journal: Comput Math Methods Med.

#### 3.7.2. Number of Cardiac Cycles Simulated

As 10 studies were performed with a constant inlet flow, the number of simulated cardiac cycles here is irrelevant. In 11 of the other 24 papers, the number of simulated cycles was specified [12, 14, 17, 18, 32, 35, 36, 38–41]. In the majority of these studies, four cardiac cycles were calculated [12, 32, 38, 39, 41]. The minimal and maximal number of simulated cycles was, respectively, one and five [14, 17].

#### 3.7.3. Time Step Size

Information on time step size for the simulation was provided in 13 papers [12, 14, 18, 30, 32, 33, 35, 36, 38–42]. The value varied between 0.0001 and 0.015 seconds per step. In three papers, only the total number of time steps was specified. This varied between 256 and 16000 time steps for four cardiac cycles [12, 38, 41]. A time-step independence test was performed in one study [40].

#### 3.7.4. Convergence Criteria

The used convergence criteria were specified in 13 papers [14, 15, 17, 19, 23, 24, 30, 35, 36, 38, 39, 42, 44]. In most of these studies, convergence criteria were set at 10*e*-4 [14, 35, 36, 38, 39]. The used convergence criteria varied between 10-3 and 10-7 [15, 42].

### 3.8. Computational Time

The computational time for the cases was described in six papers. The reported time per case varied between a couple of hours up to 1-2 months [21, 23, 35, 38, 39, 41]. In one paper, the difference in computational time for the same case with a different number of cores was shown. With the use of “supercomputers,” computational time was reduced to a couple of hours for highly complex cases [35].

### 3.9. Results and Validation

The results presented in the included papers varied according to the research question proposed. In most papers, two or three numerical outcomes were presented, i.e., pressure and WSS or streamlines and flow rates. In the majority of the papers, figures showed the results of the peak systolic and one or two diastolic time steps. Velocity and WSS were the results most reported followed by, respectively, pressure, streamlines, and flow rates. Pressure outcomes were presented either by the peak systolic numbers and energy loss over a stenosis or as the time-pressure curve over the cardiac cycle.

In nine papers, clinical data of the included patients was used to validate the CFD results (Table 4) [12, 19, 27, 32, 33, 37, 39, 40, 45]. In seven of these papers, one hemodynamic outcome was validated [12, 19, 27, 32, 33, 37, 39, 45]. These were flow results in four, pressure in two papers, and regurgitation fraction in one paper. One paper verified pressure as well as flow rate results [40]. In all the papers validating computational pressure outcomes, cardiac catheterization data was used as the golden standard. In three papers, the absolute numbers of diastolic and systolic pressure outcomes were presented and validated [12, 27, 32]. The invasively measured pressure curve was compared to the computational pressure curve in one study [40]. Other sources for validation were cardiac MRI or lung perfusion scans. With data from these sources, flow rate, flow split, and regurgitation fraction outcomes were validated. In one paper, the source of validation of the flow rates was not specified [33]. One paper verified wall deformation results of a non-patient-specific case using an experimental mock-loop setup [19]. In the 26 other papers, there was no comparison between CFD outcomes and clinical data.

The article "Computational Analysis of the Pulmonary Arteries in Congenital Heart Disease: A Review of the Methods and Results" was published in 2021. Journal: Comput Math Methods Med.

## 4. Discussion

The use of advanced imaging modalities to describe the hemodynamic impact of PA stenosis is increasing. CFD is one of these techniques providing detailed visualization of patient-specific hemodynamics. The aim of this paper was to review the numerical methods and—clinical—validation of CFD for evaluation of PA's in biventricular CHD. All of the papers included in this review emphasize the importance of hemodynamic evaluation of the PA's in biventricular CHD. They show the use and feasibility of CFD for this purpose and the wide variety of applications of the technique, i.e., for surgical or interventional treatment planning, research on complications, and exercise simulation. However, this review also shows limitations of the current available literature.

The literature reveals a large diversity in the setup for the numerical analysis of PA stenosis. This heterogeneity is important as variations in the numerical case setup significantly influence the outcomes. Results of patient-specific analysis are highly dependable on the source and quality of the anatomic reconstruction. In addition, small differences in the applied inlet or outlet boundary conditions can have a major impact. Outcomes of WSS and velocity can differ up to 30% with different boundary conditions [46–49]. In the included papers for this review, 10 different sources for anatomic reconstruction were used and 10 different methods were identified for the definition of the inlet boundary conditions. The largest variety however is seen in the definition of outlet boundary conditions. The 34 papers described 17 different approaches to assign outlet boundary conditions with very limited use of complete patient-specific boundary conditions. In the majority of cases, assumptions or generalizations defined inlet and or outlet boundary conditions. In several papers, key methodological information was missing. This included missing information on mesh size (23/34), number of cardiac cycles simulated (15/34), and convergence criteria (21/34).

The article "Computational Analysis of the Pulmonary Arteries in Congenital Heart Disease: A Review of the Methods and Results" was published in 2021. Journal: Comput Math Methods Med.

The heterogeneity, assumptions, and generalizations in the computational setup result in uncertainties regarding the outcomes. The validation of methods and results is therefore of major importance. It provides direct feedback on the used methods and increases confidence in the reliability of the technique. This review shows that the level of validation of the CFD outcomes is very low. Studies with the main aim to validate CFD outcomes were completely missing, and only nine of the 31 papers compared their outcomes to clinical data. This lowers the translational value of the studies.

Another important limitation for the clinical utility of CFD is the computational time. This was reported to be as long as several days to even months per case. However, more and more progress is made in speeding up the computational process. By use of “super computers,” improved algorithms, and cloud-based environments, the simulation time can be significantly reduced. Great examples of these efforts are shown by the two papers of Kong et al. included in this review. They show how the use of multiple cores and adjustment of algorithms can decrease computational time with several hours [35, 36]. This can be expected to further decrease in the coming years.

## 5. Conclusion

The aim of this review was to evaluate the available literature on numerical analysis of the PA's in biventricular CHD. The focus was on the used methods and the rate of—clinical—validation of the outcomes. To the best of our knowledge, this is the first review evaluating the different strategies for numerical studies of the PA's. The included literature shows the wide variety of applications of CFD and emphasizes the added value of numerical studies for hemodynamic assessment of the PA's. However, this review also shows the large heterogeneity in used methods in all parts of the numerical setup and little validation of the results. This limits the current clinical utility of CFD. To increase the translation towards clinical use, standardization of the methodologies is desirable. Future research should therefore be pointed towards validation of methods of numerical studies.

## Figures and Tables

**Figure 1:** Flowchart showing the outcomes of the literature search and inclusion and exclusion criteria. The terms used for the search were “pulmonary arteries” and “computational fluid dynamics” and their synonyms.

**Figure 2:** The different sources for reconstruction of a PA anatomy used in the included papers. (i) Gundelwein et al. 2018 [32], Kato et al. 2018 [30], Kong et al. 2017 [36], Kong et al. 2019 [35], Matthews et al. 2011 [20], Waniewski et al. 2005 [42], Zhang et al. 2020 [44], (ii) Chern et al. 2012 [39], Das et al. 2011 [40], Guibert et al. 2014 [34], Spilker et al. 2007 [12], Tang et al. 2011 [41], (iii) Ascuitto et al. 2017 [27], (iv) Berdajs et al. 2015 (1) [29], Berdajs et al. 2015 (2) [28], Chern et al. 2008 [38], Mosbahi et al. 2014 [22], (v) Lashkarinia et al. 2018 [19], Piskin et al. 2017 (2) [24], Boumpouli et al. 2020 [17], (vi) Corno et al. 2006 [13], Esmaily-Moghadam et al. 2015 [14], Migliavacca et al. 2002 [15], (vii) Zhang et al. 2016 [43], (viii) Miyaji et al. 2019 [21], Piskin et al. 2017 (1) [23], Rao and Menon 2015 [25], Yang et al. 2016 [37], Yang et al. 2017 [45], Zhang et al. 2019 [26], Tomov et al. 2019 [18], Liu et al. 2020 [31], (ix) Celestin et al. 2015 [16], and (x) Caiazzo et al. 2015 [33].

The article "Computational Analysis of the Pulmonary Arteries in Congenital Heart Disease: A Review of the Methods and Results" was published in 2021. Journal: Comput Math Methods Med.

**Table 1:** Characteristics of included papers.

Author + year	Journal	Article type	Number of geometries	Based on number of patients
Corno et al. 2006 [13]	European Journal of Cardio-Thoracic Surgery	Surgical	7	—
Esmaily-Moghadam et al. 2015 [14]	Journal of biomechanical engineering	Surgical	13	—
Lashkarinia et al. 2018 [19]	Annals of Biomedical Engineering	Surgical	5	—
Matthews et al. 2011 [20]	The Journal of Heart Valve Disease	Surgical	1	1∗
Migliavacca et al. 2002 [15]	Computer Methods in Biomechanics & Biomedical Engineering	Surgical	1	—
Miyaji et al. 2019 [21]	Interactive CardioVascular and Thoracic Surgery	Surgical	18	6
Mosbahi et al. 2014 [22]	Interactive CardioVascular and Thoracic Surgery	Surgical	1	5∗
Piskin et al. 2017 (1) [23]	Journal of Biomechanics	Surgical	12	1
Piskin et al. 2017 (2) [24]	Cardiovascular Engineering and Technology	Surgical	6	—
Rao et al. 2015 [25]	Interactive CardioVascular and Thoracic Surgery	Surgical	6	2
Zhang et al. 2019 [26]	Computational and Mathematical Methods in Medicine	Surgical	6	2
Zhang et al. 2020 [44]	Computer methods and programs in biomedicine	Surgical	6	1
Ascuitto et al. 2017 [27]	Interactive CardioVascular and Thoracic Surgery	Surgical	4	4 (3 univentricular)
Berdajs et al. 2015 (1) [29]	Journal of Surgical Research	Surgical	1	10∗
Berdajs et al. 2015 (2) [28]	Interactive CardioVascular and Thoracic Surgery	Surgical	4	20∗
Celestin et al. 2015 [16]	Pediatric Cardiology	Surgical	8	2
Kato et al. 2018 [30]	Interactive CardioVascular and Thoracic Surgery	Surgical	6	6
Tomov et al. 2019 [18]	Journal of the American Heart Association	Surgical	1	1
Liu et al. 2020 [31]	Computational and mathematical methods in medicine	Surgical	35	1
Boumpouli et al. 2020 [17]	Medical engineering and physics	Hemodynamics	9	—
Chern et al. 2008 [38]	Journal of Biomechanics	Hemodynamics	3	10
Chern et al. 2012 [39]	Computational and Mathematical Methods in Medicine	Hemodynamics	4	4
Das et al. 2011 [40]	Tech Science Press	Hemodynamics	2	2
Tang et al. 2011 [41]	Annals of Biomedical Engineering	Hemodynamics	6	6
Waniewski et al. 2005 [42]	Artificial Organs	Hemodynamics	5	1
Yang et al. 2017 [45]	Congenital Heart Disease	Hemodynamics	10	4
Zhang et al. 2016 [43]	Interactive CardioVascular and Thoracic Surgery	Hemodynamics	5	1
Guibert et al. 2014 [34]	Medical Image Analysis	Technical	17	17
Kong et al. 2017 [36]	International Journal for Numerical Methods in Biomedical Engineering	Technical	1	1
Kong et al. 2019 [35]	International Journal for Numerical Methods in Biomedical Engineering	Technical	1	1
Spilker et al. 2007 [12]	Annals of Biomedical Engineering	Technical	4	2∗∗
Yang et al. 2016 [37]	Biomechanics and Modeling in Mechanobiology	Technical	4	2
Caiazzo et al. 2015 [33]	Cardiovascular Engineering and Technology	Interventional	12	1
Gundelwein et al. 2018 [32]	Journal of Biomechanics	Interventional	32	16

∗ Animal cases ∗∗ 1 animal case, 1 human case. N/A= not applicable.

The article "Computational Analysis of the Pulmonary Arteries in Congenital Heart Disease: A Review of the Methods and Results" was published in 2021. Journal: Comput Math Methods Med.

**Table 2:** Used boundary conditions in the included articles.

Author + year	Inlet	Pulsatile	Patient specific?	Outlet	Patient specific?
Berdajs et al. 2015 (1) [22]	Mass flow	Yes	-	Pressure	-
Berdajs et al. 2015 (2) [21]	Mass flow	-	-	Pressure	-
Mosbahi et al. 2014 [20]	Mass flow	-	-	Pressure	-
Yang et al. 2016 [42]	Mass flow	Yes	In volume	Lumped parameters	Yes
Yang et al. 2017 [44]	Mass flow	Yes	In volume	Lumped parameters	Yes
Guibert et al. 2014 [25]	Mass flow	Yes	-	Lumped parameters	-
Gundelwein et al. 2018 [24]	Mass flow	Yes	In volume	Lumped parameters	Yes
Kato et al. 2018 [39]	Mass flow	Yes	In volume	Pressure	-
Zhang et al. 2016 [43]	Mass flow	Yes	Yes	Pressure	-
Zhang et al. 2020 [34]	Mass flow	-	-	Resistance	-
Rao et al. 2015 [30]	Mass flow	-	In volume	Pressure	-
Migliavacca et al. 2002 [15]	Mass flow	-	-	Pressure	-
Miyaji et al. 2019 [19]	Mass flow	-	-	Pressure	-
Spilker et al. 2007 [12]	Mass flow	Yes	For one case	Impedance	For one case
Tang et al. 2011 [41]	Mass flow	Yes	Yes	Resistance	Yes
Liu et al. 2020 [35]	Mass flow	-	-	Resistance	Yes
Kong et al. 2017 [38]	Mass flow	Yes	-	No traction	-
Corno et al. 2006 [13]	Mass flow	Yes	-	UN	UN
Piskin et al. 2017 (1) [29]	Velocity	-	-	Resistance	-
Boumpouli et al. 2020 [17]	Velocity	Yes	-	Pressure, flow split, lumped parameters	-
Chern et al. 2012 [27]	Velocity	Yes	Yes	Pressure	-
Lashkarinia et al. 2018 [36]	Velocity	-	-	Pressure	-
Kong et al. 2019 [40]	Velocity	Yes	-	No traction	-
Tomov et al. 2019 [18]	Velocity	Yes	-	Pressure	-
Waniewski et al. 2005 [33]	Velocity	Yes	-	Mass flow	-
Chern et al. 2008 [26]	Velocity	Yes	-	UN	UN
Ascuitto et al. 2017 [32]	Pressure	Yes	Yes	Pressure	Yes
Celestin et al. 2015 [16]	Pressure	-	Yes	Pressure	Yes
Caiazzo et al. 2015 [23]	Pressure	Yes	-	Lumped parameters	-
Matthews et al. 2011 [37]	Pressure	Yes	-	Pressure	-
Piskin et al. 2017 (2) [45]	Resistance	-	-	Resistance	-
Das et al. 2011 [28]	Womersley profile	Yes	Yes	Pressure/Womersley profile	Yes
Zhang et al. 2019 [31]	Lumped parameters	-	-	Lumped parameters	-
Esmaily-Moghadam et al. 2015 [14]	Lumped parameters	Yes	-	Lumped parameters	-

UN=unknown.

The article "Computational Analysis of the Pulmonary Arteries in Congenital Heart Disease: A Review of the Methods and Results" was published in 2021. Journal: Comput Math Methods Med.

**Table 3:** Validation.

Author + year	Validation of	Source validation
Ascuitto et al. 2017 [27]	Flow rates	Cardiac catheterization continuous wave Doppler
Caiazzo et al. 2015 [33]	Flow rates	UN
Yang et al. 2016 [37]	Flow split	Lung perfusion scan
Yang et al. 2017 [45]	Flow split	Lung perfusion scan
Das et al. 2011 [40]	Pressure and flow rates	Cardiac catheterization, MRI
Gundelwein et al. 2018 [32]	Pressure	Cardiac catheterization
Spilker et al. 2007 [12]	Pressure	Cardiac catheterization
Chern et al. 2012 [39]	Regurgitation fraction	CMR
Lashkarinia et al. 2018 [19]	Wall deformation	Experimental set-up

UN=unknown.

**Table 4:** Characteristics of included papers.

Author + year	Anatomy	Mesh sensitivity	Mesh element number	Inlet BC	Outlet BC	Wall compliance	Fluid rheology
Ascuitto et al. 2017 [27]	Angiography	No	UN	Pressure	Pressure	No	Newtonian
Berdajs et al. 2015 (1) [28]	Not patient-specific	No	365,000	Mass flow	Pressure	No	Newtonian
Berdajs et al. 2015 (2) [29]	Not patient-specific	No	365,000	Mass flow	Pressure	No	Newtonian
Boumpouli et al. 2020 [17]	Not patient-specific	No	90,000-125,000	Velocity	Pressure, flow split, lumped parameters	No	Newtonian
Caiazzo et al. 2015 [33]	MRI	Yes	158,000-670,000	Pressure	Lumped parameters	No	Newtonian
Celestin et al. 2015 [16]	Angiography	Yes	1,000,000	Pressure	Pressure	No	Newtonian
Chern et al. 2008 [38]	Not patient-specific	Yes	72,900	Velocity	UN	No	Newtonian
Chern et al. 2012 [39]	MRI	Yes	1,000,000	Velocity	Pressure	No	Newtonian
Corno et al. 2006 [13]	Not patient-specific	No	UN	Mass flow	UN	No	UN
Das et al. 2011 [40]	MRI	Yes	150,000-650,000	Womersley profile	Pressure/Womersley profile	No	Non-Newtonian
Esmaily-Moghadam et al. 2015 [14]	Not patient-specific	Yes	400,000	Lumped parameters	Lumped parameters	Yes	Newtonian
Guibert et al. 2014 [34]	MRI	No	UN	Mass flow	Lumped parameters	No	UN
Gundelwein et al. 2018 [32]	CT	No	60,000	Mass flow	Lumped parameters	Yes	Newtonian
Kato et al. 2018 [30]	CT	No	2,000,000	Mass flow	Pressure	No	Newtonian
Kong et al. 2017 [38]	CT	No	UN	Mass flow	No traction	No	Newtonian
Kong et al. 2019 [35]	CT	No	1,000,000	Velocity	No traction	Yes	Newtonian
Lashkarinia et al. 2018 [19]	Not patient-specific	Yes	UN	Velocity	Pressure	Yes	Newtonian
Liu et al. 2020 [31]	CT	Yes	3,723,041	Mass flow	Resistance	No	Newtonian
Matthews et al. 2011 [20]	CT	No	1,000,000	Pressure	Pressure	Yes	N/A
Migliavacca et al. 2002 [15]	Not patient-specific	Yes	30,000-48,000	Mass flow	Pressure	Yes	Newtonian
Miyaji et al. 2019 [21]	CT	No	1,000,000	Mass flow	Pressure	No	Newtonian
Mosbahi et al. 2014 [22]	Not patient-specific	No	365,000	Mass flow	Pressure	No	Newtonian
Piskin et al. 2017 (1) [23]	CT	Yes	1,007,223	Velocity	Resistance	No	Newtonian
Piskin et al. 2017 (2) [24]	Not patient-specific	Yes	1,135,156	Resistance	Resistance	No	Newtonian
Rao and Menon 2015 [25]	CT	No	UN	Mass flow	Pressure	No	Newtonian
Spilker et al. 2007 [12]	MRI	No	UN	Mass flow	Impedance	Yes	Newtonian
Tang et al. 2011 [41]	MRI	Yes	1,500,000	Mass flow	Resistance	No	Newtonian
Tomov et al. 2019 [18]	CT	Yes	>200,000	Velocity	No traction	No	Newtonian
Waniewski et al. 2005 [42]	CT	Yes	120,000-150,000	Velocity	Mass flow	No	Newtonian
Yang et al. 2016 [37]	CT	No	UN	Mass flow	Lumped parameters	Yes	UN
Yang et al. 2017 [44]	CT	No	UN	Mass flow	Lumped parameters	Yes	Newtonian
Zhang et al. 2016 [43]	CT	Yes	600,000	Mass flow	Pressure	No	Newtonian
Zhang et al. 2019 [26]	CT	No	UN	Lumped parameters	Lumped parameters	No	Newtonian
Zhang et al. 2020 [44]	CT	Yes	1,969,627	Mass flow	Resistance	No	Newtonian
